The article "Quercetin Promotes TFEB Nuclear Translocation and Activates Lysosomal Degradation of Ferritin to Induce Ferroptosis in Breast Cancer Cells" was published in 2022. Journal: Comput Intell Neurosci.

# Quercetin Promotes TFEB Nuclear Translocation and Activates Lysosomal Degradation of Ferritin to Induce Ferroptosis in Breast Cancer Cells

**DOI:** 10.1155/2022/5299218

**Published:** 2022-07-18

**Authors:** Songbo An, Mingyue Hu

**Affiliations:** Department of Pharmacy, The First People's Hospital of Lianyungang, Lianyungang, Jiangsu 222002, China

## Abstract

*Objective*. To investigate the antiproliferative efficacy of quercetin on breast cell lines and its mechanism of ferroptosis regulation. Cells (MCF-7 and MDA-231) were treated with quercetin at 0.1, 1, and 10 *μ*M, respectively. The cell counting kit-8 (CCK-8) assay was applied to assess cell viability, and the intracellular iron level, malondialdehyde (MDA), and carbonylated protein were measured. After treating the cells with quercetin, western blot was applied to determine the level of transcription factor EB (TFEB) and lysosomal-associated membrane protein 1 (LAMP-1) in cells. Meanwhile, western blot was performed to assess the nuclear translocation of TFEB protein in cells. TFEB siRNA and autophagy lysosomal inhibitor, chloroquine, were used to block ferroptosis induced by quercetin. Quercetin induced breast cancer cell death and upregulated the level of iron, MDA, and carbonyl protein in a concentration-dependent manner. Meanwhile, TFEB was highly expressed in the nucleus and lowly expressed in the cytoplasm. The high expression of TFEB promoted the expression of lysosome-related gene LAMP-1, which in turn promoted the degradation of ferritin and the release of ferric ions. The above pharmacodynamic effects of quercetin can be blocked by TFEB siRNA or chloroquine. Quercetin promotes TFEB expression and nuclear transcription, induces the onset of iron death, and thus exerts a pharmacological effect on killing breast cancer cells.

## 1. Introduction

In the female population, breast cancer is the most frequent malignancy [1]. Approximately 70–80% of patients with early-stage breast cancer can be cured [2]; however, existing treatments are not very effective for patients with advanced breast cancer [3]. The main goals of current treatment for breast cancer are to extend the lifespan of patients and to minimize the side effects of the treatment modality. The aim is to maintain or improve the quality of life of the patient. Hence, there is an urgent need to discover therapeutic drugs that can treat breast cancer with few side effects. Quercetin is a flavonoid found in plants. Quercetin is present in a variety of fruits and vegetables, such as onions, grapes, apples, and leafy greens [4]. Quercetin can inhibit the proliferation of many types of tumors. Furthermore, quercetin is involved in a number of physiological activities, such as participating in antioxidation, suppressing inflammatory responses, repressing fibrosis, and limiting viral proliferation [5–7]. The antitumor effects of quercetin can be attributed to various mechanisms, like cell cycle arrest, autophagy, and induction of endogenous and exogenous apoptotic pathways [8, 9]. Clinical chemotherapy treatments are prone to serious side effects, but oral quercetin for several months has proven to be safe and effective with no significant adverse effects [10]. However, the potential mechanism of action against breast cancer is unclear. Ferroptosis is a recently identified programmed cell death process featuring the accumulation of iron-dependent lipid peroxides [11]. Much attention has been paid to how ferroptosis affects physiological processes and various diseases. Cancer cells are more iron-dependent and more sensitive to ferroptosis than normal cells [12]. Therefore, the ferroptosis mechanism is regarded as a new novel strategy for cancer treatment. Recent research has shown that naturally active substances can promote cellular ferroptosis and eliminate multidrug resistance in cancer [13]. Some scholars have discovered a new mechanism named ferritinophagy that facilitates ferroptosis by activating the lysosomal pathway to degrade ferritin to release iron ions [14]. Lysosomes can be functionally regulated in a transcription-dependent way, such as transcription factor EB (TFEB) after nuclear transfer, which facilitates gene expression related to the regulation of lysosomal function [15]. Therefore, promoting the activation of lysosomes to degrade ferritin is a potential mechanism of antitumor drug intervention. Based on this, the object of this study was to see if quercetin might cause ferroptosis in breast cancer cell lines and to further explore its mechanism of action through the TFEB-lysosome pathway to induce ferroptosis. It provides the basis for an in-depth understanding of the anticancer mechanism of quercetin.

The article "Quercetin Promotes TFEB Nuclear Translocation and Activates Lysosomal Degradation of Ferritin to Induce Ferroptosis in Breast Cancer Cells" was published in 2022. Journal: Comput Intell Neurosci.

## 2. Materials and Methods

### 2.1. Reagents and Instruments

Quercetin and chloroquine were obtained from Sigma-Aldrich; Primary antibodies for western boltting are as follows: TFEB (Cell Signaling Technology, Danvers, MA, USA), a-tubulin (Sigma-Aldrich, St. Louis, MO, USA), LAMP-1 (Santa Cruz, Santa Cruz, CA, USA), FTL (Abcam, USA), LaminA/C (Santa Cruz, Santa Cruz, CA, USA), GAPDH (Santa Cruz); TFEB siRNA was purchased from Life Technologies. (Santa Cruz), FTL (Abcam), LaminA/C (Santa Cruz), GAPDH (Santa Cruz, Santa Cruz, CA, USA) were used in this study. TFEB siRNA was purchased from Life Technologies; Fe on assay kit, MDA assay kit, and carbonylated protein ELISA kit were purchased from Nanjing Jiancheng Biological Engineering (Nanjing, China). The cytoplasmic cytosolic protein extraction and isolation kits were purchased from Beyotime (Beijing, China). Breast cancer cell lines were sourced from the National Collection of Authenticated Cell Cultures.

### 2.2. Cell Culture

Breast cancer cell lines were cultured and grown in Dulbecco's Modified Eagle Medium (DMEM) containing 10% FBS. Breast cancer cells were planted in 6-well or 96-well plates and treated for 24 hours with 0.1, 1, and 10 M quercetin. TFEB siRNA transfection was performed using DharmaFECT 4 transfection reagent (Dharmacon). The effect of protein silencing was detected by western blot.

### 2.3. CCK-8 Assay

Single cell suspension was added uniformly to a 96-well plate (100 *μ*L/well). After 24 h, 10 uL CCK-8 mixture was prepared and added to the wells and the cells were incubated. Cells and CCK-8 solution were incubated for 4 h. The absorbance value of each well was detected at 450 nm using a microplate reader.

### 2.4. Determination of Ferroptosis Indicators

First, according to the commercial kit instructions, the kits should be withdrawn from the refrigerator 1 hour before the experiment to allow all the reagents to return to room temperature for more stable results. Second, after cell culture, cell lysates were extracted and intracellular levels of MDA, iron, and glutathione (GSH) were assayed using biochemical reagents according to the instructions of commercial kits. The carbonylated protein content was determined using enzyme-linked immunosorbent assay (ELISA) kits.

### 2.5. Cytoplasmic Cytosolic Protein Extraction

After treatment of MCF-7 cells, wash with PBS and incubate with Cytoplasmic Extraction Reagent I for 10 min, and then treat with precooled Cytoplasmic Extraction Reagent II. After centrifugation at 12,000*g* for 5 min, the supernatant was collected. The insoluble fraction is resuspended in prechilled Nuclear Protein Extraction Reagent for 40 min and then centrifuged at 12,000*g* for 10 min. The supernatant was immediately extracted as a nuclear protein extract. BCA was used to determine the protein content. The samples were kept at −80°C.

### 2.6. Western Boltting Detecting the Protein Expression of TFEB, FTL, and LAMP-1 in MCF-7 cells

Cell lysis buffer containing 0.5% protease inhibitor was used to lyse MCF-7 cells. The bicinchoninic acid (BCA) kit was used to perform protein concentration. To perform electrophoresis, equal amounts of protein samples (40 mg) were placed in a 10% gel and the proteins were transferred to a PVDF membrane. After 1 hour of blocking with 5% nonfat milk in TBST. The membranes were treated with primary antibodies overnight at 4°C before being incubated with HRP-conjugated secondary antibodies for 1 hour at room temperature. An enhanced chemiluminescence (ECL) test kit was used to detect the target protein. ImageJ was used to perform quantitative analysis on all of the data.

The article "Quercetin Promotes TFEB Nuclear Translocation and Activates Lysosomal Degradation of Ferritin to Induce Ferroptosis in Breast Cancer Cells" was published in 2022. Journal: Comput Intell Neurosci.

### 2.7. Statistical Analysis

The data were presented as mean SD (*n* = 5), and the Shapiro–Wilk test was used to determine normality. Student's *t*-test was used to compare statistical differences between the two groups. Multiple group comparisons were carried out using one-way or two-way ANOVA, followed by Bonferroni's post hoc test (only when *P* < 0.05). GraphPad Prism 7.0 was used for all statistical analyses.

## 3. Results

### 3.1. Quercetin Promotes Ferroptosis in Breast Cancer Cells

MCF-7 and MDA-MB-231 cells were tested for vitality after being treated with the ferroptosis inducers erastin and quercetin. Erastin caused a dramatic decrease in cell activity compared to the control group (*P* < 0.001). The cell viability of MCF-7 and MDA-MB-231 was decreased after treated with 10 *μ*M quercetin (Figure 1(a)). As shown in Figure 1(b), erastin increased intracellular iron ion level significantly. In addition, as the concentration of quercetin increased, the intracellular iron ion content also increased accordingly. In MCF-7 cells, the quercetin-induced decrease in cell viability and increase in iron ion content were more pronounced (*P* < 0.001). MCF-7 cells may be more susceptible to ferroptosis, according to the results of the study. The expression of intracellular malondialdehyde (MDA) and carbonylation protein (CFP) gradually increased with longer treatment time of quercetin, revealing that quercetin inhibited breast cancer cell development by causing ferroptosis.

### 3.2. Quercetin Promotes TFEB Nuclear Translocation and Lysosomal Activation-Related Gene Expression in Breast Cancer Cells

MCF-7 cells were exposed to 10 mM quercetin for 0, 6, and 12 h, and the intracellular distribution of TFEB was observed by extracting cellular plasma and cellular nuclear proteins. Figures 2(a) and 2(b) demonstrate that the nuclear translocation of TFEB was evident after 6 h of quercetin treatment. After 12 hours of quercetin treatment, TFEB was further transferred into the nucleus, and at this time, TFEB was basically located in the nucleus with less expression in the cytoplasm. At 12 h, the nuclear translocation was highly considerable (*P* < 0.001) compared to 0 h, indicating that quercetin can promote nuclear transcription of TFEB. Later, MCF-7 was treated with quercetin for different times. The intracellular expression of TFEB increased with the increase of quercetin treatment time, and the highest expression was observed at 24 h. It showed that quercetin could promote the nuclear transcription of TFEB in the cells and also act by increasing protein expression. LAMP-1, one of the lysosome-related proteins, is transcriptionally regulated by TFEB, and its intracellular content gradually increased with the prolongation of quercetin stimulation. It is suggested that quercetin can promote the expression of lysosome-related genes by regulating the expression of TFEB and nuclear transcription.

The article "Quercetin Promotes TFEB Nuclear Translocation and Activates Lysosomal Degradation of Ferritin to Induce Ferroptosis in Breast Cancer Cells" was published in 2022. Journal: Comput Intell Neurosci.

### 3.3. Quercetin Regulates TFEB to Promote Lysosomal Release of Iron Ions

To make sure if quercetin promotes ferroptosis in breast cancer cells by controlling TFEB activation of lysosomes, resulting in higher intracellular iron ion levels, in this study, first, we verified that TFEB siRNA could effectively knock down TFEB in MCF-7 cells (Figure 3(a)). The intracellular ferritin content was reduced after quercetin treatment (*P* < 0.001), and quercetin-induced ferritin degradation was inhibited after achieving TFEB gene silencing (*P* < 0.001). Similarly, the use of chloroquine, a lysosomal function inhibitor, also inhibited quercetin-induced ferritin degradation (*P* < 0.001) (Figure 3(b)). Meanwhile, the use of either TFEB siRNA or chloroquine resulted in an increase in quercetin-induced intracellular ferric ion content (*P* < 0.001) (Figure 3(c)). In contrast, cell viability decreased with quercetin treatment, while both TFEB siRNA and chloroquine could block the lethal effect of quercetin on breast cancer cells (*P* < 0.001) (Figure 3(d)). According to the above data, quercetin exerts its lethal effect on breast cancer cells by promoting TFEB transcription to activate lysosomal degradation of ferritin, promoting the elevation of intracellular ferric ion content, and inducing the onset of cellular feroptosis (Figure 4).

## 4. Discussion

Quercetin is increasingly being used as a nutrient to boost immunological response and circulatory system fitness [16]; however, its potential for anticancer applications remains unclear. Our study showed that quercetin induced the death of various breast cancer cells. Further studies suggest that the mechanism of breast cancer inhibition by quercetin may be related to the promotion of lysosomal activation mediated by TFEB and subsequent ferritin degradation. The degraded ferritin subsequently releases large amounts of ions, which ultimately promote iron-dependent lipid peroxidation and ferroptosis. These findings are significant for further research into the possible use of quercetin in clinical cancer therapy.

Autophagy can degrade cellular contents via the lysosomal pathway, and therefore modulation of autophagy is increasingly considered an effective strategy for anticancer therapy [17]. Quercetin-induced cell death can be effectively prevented by the use of the autophagy lysosomal inhibitor chloroquine. This difference makes lysosomal activation a key potential mechanism of quercetin-induced cell death.

The article "Quercetin Promotes TFEB Nuclear Translocation and Activates Lysosomal Degradation of Ferritin to Induce Ferroptosis in Breast Cancer Cells" was published in 2022. Journal: Comput Intell Neurosci.

We found that quercetin can increase lysosomal ferritin breakdown by increasing TFEB nuclear translocation and lysosomal gene transcriptional activation. Lysosomes play a crucial role in the integrity of the intracellular environment, and in addition to their degrading function, they also act as an important signal transducer and are involved in a range of physiological functions [18]. The significance of lysosomes in cancer is complicated and hotly debated. It has been found that removing TFEB from cells can protect them from clomiphene-induced cell death [19]. However, another study found that activating TFEB improves lysosomal function and reduces doxorubicin-induced apoptosis [20]. These contentious investigations may yield contradictory results based on the different stimulation parameters and cell lines used. They all, however, stress the necessity of targeting the TFEB-lysosomal pathway as a feasible anticancer therapy.

Lysosome-dependent cell death is caused by increased permeability or rupture of the lysosomal membrane, and this damage eventually leads to histone leakage, which activates cysteine cleavage and triggers apoptosis through protein hydrolysis [21]. However, lysosomal inhibitors were used in this study to prevent quercetin-induced cell death, suggesting that cell death promoted by quercetin results from activation of lysosomal function rather than from disruption of the structure of the lysosome. According to previous studies, ferritin accumulates in lysosomes and co-localizes with autophagy-associated (ATG) proteins [22]. The induction of autophagy is required for the activation of ferroptosis, and the degradation of lysosomal ferritin is a specific type of autophagy that contributes to the onset of iron toxicity [23]. Cells can utilize the free iron produced by lysosomes to make lipoxygen as a consequence of ferritin lysosomal degradation. After a series of signaling, quercetin eventually triggers the release of iron ions, leading to cellular ferroptosis. Ion homeostasis is critical for cell survival because excess free iron is hazardous, causing oxidative stress and cell death, including ferroptosis [24]. Alternatively, lysosomal inhibition may isolate iron in the lysosome, resulting in the inability of cells to access iron and thus inhibiting ferroptosis from occurring. This disparity can also be attributed to the tolerance of different cell types to iron levels. Iron levels in cancer cells are higher than those in noncancerous ones, according to accumulating data. Therefore, iron-targeting therapeutic effects of quercetin are practical in clinical cancer treatment and prevention.

The article "Quercetin Promotes TFEB Nuclear Translocation and Activates Lysosomal Degradation of Ferritin to Induce Ferroptosis in Breast Cancer Cells" was published in 2022. Journal: Comput Intell Neurosci.

## Figures and Tables

**Figure 1:** Quercetin promotes ferroptosis in breast cancer cells. (a) The CCK-8 assay was applied to detect the cell proliferation. (b) Iron ion detection kit was used to detect the content of iron in cells. (c) MDA kit was used to detect intracellular MDA content. (d) The ELISA kit was used to detect the expression of carbonylated protein. ^*∗*^*P* < 0.05, ^*∗∗*^*P* < 0.01, and ^*∗∗∗*^*P* < 0.001.

**Figure 2:** Quercetin promotes TFEB nuclear translocation and lysosomal activation-related gene expression in breast cancer cells. (a, b) Detection of TFEB protein distribution by western blotting. (c, d) MCF-7 cells were treated with 10 *μ*M quercetin for 0, 1, 4, 8, 12, and 24 h and the protein expression of TFEB and LAMP-1 was detected by western blotting. ^*∗*^*P* < 0.05, ^*∗∗*^*P* < 0.01, and ^*∗∗∗*^*P* < 0.001.

**Figure 3:** Quercetin regulates TFEB and promotes the release of iron ions from lysosomes. (a) MCF-7 cells were treated with NC or TFEB siRNA, respectively, and TFEB protein expression level was detected. MCF-7 cells were incubated with quercetin, TFEB siRNA, and chloroquine alone or co-incubated to detect intracellular ferritin expression (b), iron ion levels (c), and cell viability (d). ^*∗*^*P* < 0.05, ^*∗∗*^*P* < 0.01, and ^*∗∗∗*^*P* < 0.001.

**Figure 4:** The mechanism of quercetin-induced ferroptosis in breast cancer cells.

## Data Availability

The datasets used and analyzed in this study are available from the corresponding author on reasonable request.
